# Isolated Superior Mesenteric Artery Dissection After Methamphetamine Use: A Rare Adverse Effect

**DOI:** 10.7759/cureus.19551

**Published:** 2021-11-13

**Authors:** Rayan A Alzahrani, Omar M Alzahrani, Sarah H Alherz, Abdulrahman A Alzahrani, Omran M Alzahrani, Mohammed A Alqarni, Khalid Abdulrahman A Alzahrani, Khalid Abdulkarim H Alzahrani, Suhayb A Al Zahrani, Abdulaziz A Alzahrani, Hamad A Alghamdi, Malak Alshammari

**Affiliations:** 1 College of Medicine, Al-Baha University, Al-Baha, SAU; 2 College of Medicine, Imam Abdulrahman Bin Faisal University, Dammam, SAU

**Keywords:** case report, computed tomography, methamphetamine use, artery dissection, superior mesenteric artery, abdominal pain

## Abstract

Methamphetamine is the second most commonly abused drug worldwide. It is a sympathomimetic agent that works by inhibiting the reuptake of monoamine neurotransmitters, including dopamine, norepinephrine, and serotonin. Methamphetamine use is associated with early mortality, and cardiovascular complications are the leading cause of increased mortality. We discuss the case of a 41-year-old man who presented to the emergency department with a sudden abdominal pain of eight hours' duration. The pain was located in the epigastric area with radiation to the back. Upon examination, the patient appeared agitated and diaphoretic. His pupils were dilated bilaterally. His vital signs included tachycardia (120 bpm), tachypnea (24 bpm), hypertension (150/90 mmHg), and normal temperature (36.9 ℃). Abdominal examination revealed a soft and lax abdomen with no tenderness. His bowel sounds were normal. Given the physical signs, a toxicology screen was conducted and was positive for methamphetamine use. The patient reported that he used recreational drugs occasionally and admitted that the abdominal pain developed a few hours following methamphetamine use. The patient was treated with fluid resuscitation, analgesic, antihypertension medications, and anticoagulant therapy. The patient had significant improvement in his condition within 48 hours with complete resolution of the abdominal pain. Isolated superior mesenteric artery dissection is a very rare clinical condition. This case report highlights the importance of recognizing the cardiovascular adverse effects that may develop after methamphetamine use.

## Introduction

Methamphetamine is the second most commonly abused drug worldwide, after cannabis [1]. It is estimated that over 4.5 million individuals in the United States have tried methamphetamine during their lives [2]. Methamphetamine is a sympathomimetic agent that works by inhibiting the reuptake of monoamine neurotransmitters, including dopamine, norepinephrine, and serotonin. It has a variety of stimulant, euphoric, anorexiant, and hallucinogenic effects. It is reported that methamphetamine accounted for over 90,000 visits to the emergency department in the United States in 2005 [3]. The use of methamphetamine is associated with early mortality, and cardiovascular complications are the leading cause of increased mortality [4]. However, studies examining the cardiovascular complications arising from methamphetamine use have been scarce. Tachycardia and hypertension are commonly associated with patients intoxicated with methamphetamine. The reported life-threatening cardiovascular complications include arrhythmias, myocardial infarction, stroke, aortic dissection, and cardiomyopathy. Swalwell and Davis [5] conducted an autopsy study on patients who had died from aortic dissection with particular emphasis on the role of drugs. Interestingly, they found that drugs constituted the risk factor in over 40% of cases and methamphetamine was the second most common drug involved. In this report, we present the case of a middle-aged man with an isolated superior mesenteric artery dissection following methamphetamine use.

## Case presentation

Our patient was a 41-year-old man who presented to the emergency department with a sudden abdominal pain of eight hours' duration. The pain was located in the epigastric area with radiation to the back. The pain was constant and was stabbing in nature, and it was associated with nausea and vomiting. He reported that the pain worsened when lying flat on his back and was partially relieved when he leaned forward. Before the onset of his pain, the patient had been feeling well. There was no history of anorexia, weight loss, fever, or change in bowel or urinary habits. The past medical history of the patient was remarkable for well-controlled hypertension and diabetes mellitus. His medication included amlodipine 5 mg and metformin 1000 mg, and he reported good compliance with his medications. He had not undergone any previous surgery. He had a smoking history of 20 pack-years and reported no alcohol consumption. The family history was significant for ischemic heart disease.

Upon examination, the patient appeared agitated and diaphoretic. His pupils were dilated bilaterally. His vital signs included tachycardia (120 bpm), tachypnea (24 bpm), hypertension (150/90 mmHg), and normal temperature (36.9 ℃). His oxygen saturation was 99% on room air. Abdominal examination revealed a soft and lax abdomen with no tenderness. His bowel sounds were normal. Cardiorespiratory examinations were also normal. Initial laboratory investigations revealed a hemoglobin level of 14.5 g/dL, leukocytes count of 11,000/μL, and platelets count of 375,000/μL. Both serum amylase and lipase were within the normal limits. The biochemical investigation, including hepatic and renal profiles, was normal (Table 1). Given the physical signs of the patient, a toxicology screen was conducted, which was positive for methamphetamine use. The patient reported that he used recreational drugs occasionally and he admitted that the abdominal pain developed a few hours following methamphetamine use.

**Table 1:** Summary of the laboratory findings

Laboratory investigation	Unit	Result	Reference range
Hemoglobin	g/dL	14.5	13.0–18.0
White blood cell	1000/mL	8.2	4.0–11.0
Platelet	1000/mL	380	140–450
Erythrocyte sedimentation rate	mm/hr	12	0–20
C-reactive protein	mg/dL	8.2	0.3–10.0
Total bilirubin	mg/dL	0.8	0.2–1.2
Albumin	g/dL	3.5	3.4–5.0
Alkaline phosphatase	U/L	55	46–116
Gamma-glutamyltransferase	U/L	21	15–85
Alanine transferase	U/L	18	14–63
Aspartate transferase	U/L	20	15–37
Blood urea nitrogen	mg/dL	9	7–18
Creatinine	mg/dL	0.9	0.7–1.3
Sodium	mEq/L	135	136–145
Potassium	mEq/L	3.6	3.5–5.1
Chloride	mEq/L	105	98–107

Initial abdominal radiograph revealed normal findings (Figure 1). The patient underwent a CT scan of the abdomen with intravenous contrast, which demonstrated an isolated dissection involving the proximal segment of the superior mesenteric artery (Figure 2). The bowel loops were unremarkable with no evidence of ischemia. The vascular surgery team was consulted. Since the patient was hemodynamically stable, a conservative approach was taken. The patient was treated with fluid resuscitation, analgesics, antihypertension medications, and anticoagulant therapy. Within 48 hours, the patient had significant improvement in his condition with complete resolution of the abdominal pain. He received extensive counseling about his recreational drug use and agreed to enroll in a rehabilitation program. The patient was discharged on the fifth day of admission.

**Figure 1:** Plain abdominal radiograph of the patient on presentation showing no abnormalities

**Figure 2:** Sagittal image of abdominal CT angiography demonstrating dissection of the superior mesenteric artery (arrow) CT: computed tomography

## Discussion

We reported the case of a middle-aged man with isolated superior mesenteric artery dissection presenting with acute abdominal pain. To the best of our knowledge, this is the first reported case of superior mesenteric artery dissection in association with methamphetamine use. Isolated superior mesenteric artery dissection is a very rare condition with few reported cases in the literature. The first case of isolated superior mesenteric artery dissection was reported by Bauersfeld in 1947 [6]. Since then, a large number of cases have been reported thanks to the widespread use of advanced radiological imaging.

While no pathological cause is identified in most cases with isolated superior mesenteric artery dissection, the reported risk factors include atherosclerosis, cystic medial degeneration, fibromuscular dysplasia, and trauma [7]. In the present case, we believe that the stress of the arterial wall related to hypertension was the most likely contributing factor. Regarding the clinical manifestation of isolated superior mesenteric artery dissection, acute abdominal pain is the most common presentation, which may be related to the dissection itself or the resultant bowel ischemia. However, the dissection may be asymptomatic and diagnosed incidentally on imaging.

As in our case, the diagnosis of isolated superior mesenteric artery dissection can be reached by an abdominal CT angiography scan. It is crucial to evaluate the patency of the dissected artery and the presence of complications, including hematoma and bowel ischemia [8]. In the present case, there was no evidence of bowel ischemia and the artery was patent. Doppler ultrasound scan may also aid in diagnosing the superior mesenteric artery dissection but it has an inferior accuracy.

Given its rarity, there are no available treatment guidelines for an isolated superior mesenteric artery dissection. A retrospective review by Gobble et al. [7] revealed that a conservative non-operative approach may be successful in approximately half of the cases. The non-operative approach includes bowel rest and anticoagulation. Operative approaches can be performed by open surgery or an endovascular procedure. In the present case, a non-operative approach was employed with close observation for the signs of bowel ischemia.

## Conclusions

Isolated superior mesenteric artery dissection is a very rare clinical condition. This case report highlights the importance of recognizing the cardiovascular adverse effects that may develop after methamphetamine use. CT angiography can make the diagnosis accurately. If no evidence of complications is present, patients may be managed conservatively with bowel rest and anticoagulation with close observation.
